The article "The Promoting Effect of Mental Health Education on Students' Social Adaptability: Implications for Environmental" was published in 2022. Journal: J Environ Public Health.

# The Promoting Effect of Mental Health Education on Students' Social Adaptability: Implications for Environmental

**DOI:** 10.1155/2022/1607456

**Published:** 2022-06-29

**Authors:** Ying Jin

**Affiliations:** School of Physical Education & Health, Wenzhou University, Wenzhou, Zhejiang Province, China

## Abstract

Students' mental health has always been a hot topic in colleges and universities. How to make students integrate into the collective and society faster and better is also one of the most difficult problems for educators. Students want to improve their competitiveness; not only must they have superb professional skills, but at the same time, they must have good social adaptability. Only in this way can they quickly complete their identity change and quickly adapt to workplace life. Students' social adaptability is not innate, but gradually formed through long-term positive mental health education. Considering the relationship between psychoeducation and social adaptability, in general, a good psychoeducation system is conducive to the development of students' social adaptability, and they promote each other. Good mental health education is multifaceted and sustainable for the development of social adaptability. In this context, it is necessary to formulate a targeted positive mental health education plan according to the actual situation of students, so as to comprehensively improve the comprehensive quality of students in this way.

## 1. Introduction

In the context of the new era, education includes not only skills teaching, but also psychological teaching, and its teaching purpose is to cultivate all-round development talents. Positive mental health education aims to maintain students' mental health and guide students to view social phenomena from multiple perspectives. Mental health education is based on the laws of students' physical and psychological development, using psychological education methods to cultivate students' good psychological quality and promote the overall improvement of students' overall quality. Mental health education is an important part of quality education: it is an important link in implementing the “21st Century Education Revitalization Action Plan,” implementing the “Cross-century Quality Education Project,” and cultivating high-quality talents across the century. At the same time, it is also an inevitable requirement of modern education and a common urgent task faced by the majority of school educators to effectively carry out mental health education for students. In the past 20 years, the mental health of students has attracted much attention from the society. Looking back on the relevant investigation and research on students' mental health, psychological problems have often appeared. Because of the high expectations of the family, the pressure faced by students is significantly higher than that of other groups of the same age, and suicide has become the number one killer of students. In recent years, the psychological problems of students have become more and more serious. In particular, schools generally report that more and more students have problems such as poor adaptability, anxiety, and depression [1]. Mental health will have character defects, emotional defects, psychological defects, and abnormal psychology.

Students will face huge employment pressure when they are approaching graduation. To improve their employment competitiveness, it is necessary to ensure that students have a certain understanding of social development trends and can quickly adapt to the pace of social life. Looking at this issue from the perspective of schools, school administrators need to pay enough attention to mental health education and, through positive mental health education, help students develop a correct world outlook, outlook on life and value orientation, and at the same time carry out a comprehensive social development. They need to understand and help students successfully complete their identity transition. Mental health education goal is to cultivate good character quality, develop intellectual potential, enhance psychological adaptability, stimulate inner motivation, maintain mental health, and develop good behavior habits, that is, fertility, enlightenment, strength, motivation, health, and guidance. In the specific teaching process, school managers and teachers need to conduct in-depth analysis of various problems exposed in the teaching process of positive mental health education and formulate efficient mental health education teaching strategies based on the actual situation of the school [2].

## 2. State of the Art

### 2.1. Educational Goals

The adaptive goal mainly focuses on the students' present, so that students can understand the changing trends and characteristics of the future society, help them establish a long-term and stable outlook on life, values, and world outlook in line with the direction of social progress, and pursue high-level life meaning and guide them through various abilities. To cultivate students to have a correct understanding of the society around them, maintain a harmonious and good adaptive relationship with the society, make college students dare to face the reality and the future, have the courage to practice, have a quick mind, constantly revise those unrealistic fantasies, improve setback tolerance, and be fully psychologically prepared and strong, they must adapt to meet the rapidly changing society. This goal is the main task of current mental health education [3].

The developmental goal mainly focuses on the future of students. It is to take all students as the object of mental health education. It is aimed at students at different stages, at all levels, in various disciplines, and in special groups. For example, new students face weak social skills and appear interpersonal. The relationship is tense and the learning ability is weak, which causes learning difficulties. The lack of self-care ability in life results in overdependence and lack of self-awareness ability, so they cannot treat themselves correctly. Graduates face employment choice problems, interpersonal communication problems, emotional problems, and other “developmental” problems. Through developmental psychological education, students can obtain optimal and most effective development on the basis of adaptation, cultivate innovative consciousness, and enhance students' self-psychological education ability to solve various developmental problems faced by college students in their development [4]. This goal is the focus of mental health education in colleges and universities and represents the main direction of mental health education in the future. In short, in the implementation of mental health education, we should pay attention to all students as the service object and combine the three goals of mental health education to make mental health education play its due role. At the same time, with the deepening of the understanding of mental health education and the summary of practical experience, more and more people realize the importance of mental health education in colleges and universities to the growth and development of every student. The future development trend of mental health education will be towards development and growth, prevention, and treatment supplemented by the direction of development.

### 2.2. The Internal Principle of Mental Health Education to Improve Students' Social Adaptability

Students are in the final stage of formation of outlook on life and value orientation. At this stage, positive mental health education for students can guide students to form correct values, have a sound personality, quickly adjust their mentality after entering the society, and successfully complete identity conversion [5]. In addition, in order to improve their employment competitiveness, students will focus most of their energy on how to improve their professional skills, and schools and teachers also pay more attention to the level of students' professional ability. Development will have a certain impact, causing students to fall into a state of semiclosed heart, and then gradually lose their social ability. After entering the workplace, they cannot communicate well with colleagues. It is easy to have friction with leaders and colleagues at work, affecting personal development. To solve this problem, it is necessary to carry out positive mental health education for students, improve their social skills and social adaptability, and enable students to better integrate into social life.

There are many factors for judging students' comprehensive ability. In addition to the professional skills that students have mastered, good psychological quality, communication skills, and social experience are also very important factors. Through positive mental health education, students realize that only having good professional knowledge cannot improve their comprehensive competitiveness, but they have to comprehensively improve their abilities based on professional skills. Especially for some students with poor foundation, they can explore their strengths through positive mental health education, correct their attitude, and correctly examine their own advantages, so as to make up for their deficiencies in professional knowledge and ability and improve their employment competitiveness.

Innovation is an important driving force for social and economic development, and both technological innovation and theoretical innovation can expand a huge space for development. Students are active in thinking and have great potential for innovation. In the process of learning, they can improve their rational thinking ability by accepting scientific and systematic positive mental health education and learn to look at them from different perspectives (personal and social) with materialistic and dialectical thinking. For social development, summarize the law of industry development and flexibly adjust the learning plan and learning goals based on this.

Students who integrate into the society will face enormous pressures from work, life, and other aspects. If they want to keep a clear mind under tremendous pressure, they need to have strong psychological quality and ability to resist pressure. This kind of antistress ability cannot be cultivated by professional knowledge teaching. It must undergo positive mental health education, so that students can realize the multifaceted nature of social life, maintain an optimistic spirit in the face of pressure and setbacks, and quickly adjust their psychology. Once you find that you cannot carry out effective psychological construction, you should take the initiative to seek the help of a professional psychologist to help yourself get rid of the influence of negative emotions as soon as possible.

### 2.3. Factors Affecting the Mental Health of College Students

Social factors are the determinants that affect the psychological development of college students. Marxism believes that the essential attribute of man is social. Man is a social man. The process of growth in life is actually a process of socialization. Socialization is the process in which people become qualified members of society with independent personalities through interaction with the social environment under specific social material and cultural conditions [6]. For college students who are in the midst of social change, with the expansion of college enrollment and the reform of the national distribution system, this is a test of their psychological quality and comprehensive quality. Facing the society's requirements for talents, the college students are confused in their hearts, and some of the college students who do not adapt well to the society have psychological obstacles such as anxiety and depression. At the same time, the negative effects brought about by social changes, such as corruption, unhealthy ideology, and poor social facilities, will make college students unable to face and eliminate the limitations of their own knowledge, experience, and self-cultivation troubled. In addition, due to the popularization of the Internet and the wide and rapid dissemination of information, college students, as the most active, sensitive, and knowledgeable people in the society, often feel the changes and shocks first. Generally speaking, the psychological development level of the period is becoming mature but not really mature, so it is inevitable to feel confused, empty, depressed, and at a loss in the face of such changes and shocks. The main source of stress for contemporary college students is study and work, and they are under a lot of pressure at work, as shown in Figure 1.

College students spend most of their lives at school. The growth and development of college students are inseparable from school education and management. Because of the close relationship between college students and schools, the mental health of college students will inevitably be affected by school factors. At present, the main factors affecting the mental health of college students in college life are psychological discomfort caused by changes in the environment and roles; simple teaching methods cannot meet the requirements of students' study and life, which is one-sided implementation of educational ideas [7]. The emphasis on grades, ignoring ability and intellectual factors, ignoring nonintelligence factors, lack of a good interpersonal environment for college students to communicate properly with classmates and teachers, and the influence of unhealthy campus culture all have a certain impact on the development of students' mental health.

The family is the cell of society and the first social environment a person comes into contact with. Although college students are far away from their parents, the ups and downs of the family will affect the mood of college students because of the blood relationship, economic connection, and emotional maintenance. Especially in most one-child families, due to the overindulgence of their parents, they must first cultivate their self-care ability and learn to get along with others harmoniously after entering university. If these problems are not solved well, it is easy to induce psychological problems. Also from an economic point of view, poor college students with low family economic level are psychologically prone to have low self-esteem and lack of confidence [8, 9]. Poor family relationships or unsound family structures often make it difficult for college students to communicate with their families normally in emotional and other aspects and cannot meet the normal sense of belonging and love needs of college students, resulting in great psychological pressure mental disorder.

The mental health of college students is closely related to their psychological quality and psychological endurance. The same life events often have different meanings for different college students and thus have different effects on mental health. Generally speaking, the crisis of identity, the defect of personality, the incompleteness of psychological quality, and the instability of emotional development will cause different college students to adopt different attitudes towards the same thing and thus have different effects on their mental health. In the face of success and failure, how to actively control the self and adjust the self has become an important factor in preventing depression and interpersonal relationships; college students' understanding and acceptance of the physiological self and physiological diseases will affect their mental health [10]. At present, with the increase of stress and pressure brought about by the increase of stressful stimuli in the whole society, the psychological quality of college students cannot keep up with the requirements of the times fail. Once the environment becomes different from the previous one, there will be a sense of frustration; especially when the relative intensity of the setback is greater or the duration is longer, it will turn to disappointment and low self-esteem and they will become discouraged and lethargic.

## 3. The Current Mental Health Situation of Students

According to the survey data in 2020, we can see the depression tendency of current college and undergraduate students, as well as the depression status of adults in the country, as shown in Table 1.

A comprehensive analysis of the student group shows that 76.3% of the current students are in a mentally subhealthy state, only 10.3% of the students are in a normal state of mind, and 16.3% of the students have different degrees of psychological problems. It is very necessary, and the specific data is shown in Figure 2.

The specific relationship between their mental health states is shown in Figure 3. The main manifestations of their psychological problems are anxiety, hostility, paranoia, depression, etc., as shown in Figure 4.

Regarding the statistical analysis of the obtained data according to gender classification, comparing the differences between men and women, we can see that there is a certain gap in the mental health status of different genders. Women's mental health index is higher, and men are slightly more depressed than women. For details, see Figure 5.

The survey found that the current sources of psychological problems mainly include emotions, parent-child relationship, peer relationship, learning, and many other aspects, among which the repressed emotions from learning are an important factor for the student group, and the current learning pressure leads to a certain degree of psychological problems in students; the specific data is shown in Figure 5.

## 4. Mental Health Education Methods

Mental health education is different from ideological and political education, the necessity of its existence is self-evident, and it is also different from ideological and political education in the process of education and teaching; see Table 2.

### 4.1. Enrich Teaching Content

Enriching teaching content aiming at the single problem of mental health education content in colleges and universities, school administrators, and teachers should try to update and enrich the teaching content [11]. On the one hand, it is necessary to flexibly adjust the teaching structure, and add some new elements according to the social development trend, such as “comparative research on different ideas in the context of economic globalization” or “be alert to the influence of “color revolution” on young people's thinking,” so as to make mental health better. The educational content is more in line with the reality [12]. On the other hand, when teachers carry out teaching design work, they need to update the cases in the teaching plan, select some cases that are closely related to students, and make students aware of the important role of mental health education. The current basic process of psychological education activity courses is as shown in Figure 6.

There are certain differences in students' satisfaction with the current mental health education, and there is a certain understanding of the current education and teaching methods. The specific satisfaction is shown in Figure 7.

### 4.2. Clarify the Teaching Object

Positive mental health teaching is a systematic educational discipline. The goal of learning is not only to help students overcome psychological problems, but also to focus on how to improve students' psychological potential and help students build a sound personality and a strong heart. Only in this way can students calmly cope with various challenges and pressures in social work [13]. In this context, teachers should clarify the objects of mental health teaching and expand the scope of teaching, not only to carry out mental health education for students with psychological problems, but also to carry out positive mental health education for ordinary students. Treat students equally, do not evade various psychological problems raised by students, understand the real psychological state of each student through active communication, and formulate different education plans to improve teaching efficiency. In addition, in order to improve teaching efficiency, teachers should make full use of various resources, use information technology to form a complete communication system among students, schools, teachers, parents, and social enterprises, and give full play to the advantages of various resources so that students can selectively receive positive mental health education to improve their psychological quality and social adaptability.

### 4.3. Carry Out Teaching Practice

In view of the disconnection between theoretical teaching and social practice, teachers and school administrators need to actively expand teaching practice. While carrying out theoretical teaching, students have the opportunity to apply theoretical knowledge in practice. If there is a lack of practical activities, the positive psychological knowledge learned by students will not be able to play its role, nor will it achieve the goal of improving students' social adaptability. It should be noted here that the practical activities related to mental health knowledge are not unique. In short, it is not possible to set up a practical course for mental health teaching. Let the students summarize the experience in the practice process of the professional course, then analyze the students' summary from the perspective of positive psychological education, and point out which problems in the practice process are caused by the lack of positive and healthy psychology. In this way, students can be aware of the important role of positive psychological education [14–17].

### 4.4. Special Education Activities for Career Selection

Bandura's ternary interaction theory considers people's psychological activities and environmental performance from the interactive relationship between the environment, individuals, and their behaviors and regards people's psychological activities as the interaction between the environment, individuals, and their behaviors. There is two-way influence of social environment and people's internal psychological factors. As the unique environmental education force of the school, campus activities are the potential courses for students' growth. The role of a good and strong campus cultural atmosphere and diverse and effective campus activities in school education is immeasurable and cannot be replaced by any explicit curriculum and rules and regulations. As an environmental education force, it has a psychological impact and behavioral constraints on students' psychological feelings, psychological experience, psychological development, and even their learning, life, communication, and growth [18]. In accordance with the spirit of the relevant documents of the Ministry of Education, and in accordance with the requirements of the local education authorities and human resources and social security departments, organize students to carry out a series of special competitions to improve their psychological quality and vocational skills, such as career planning and design competitions, entrepreneurship design competitions, and vocational skills and competitions; invite human resources market managers, elites of enterprises and institutions, outstanding graduate representatives, etc. to come to the school to give career guidance lectures; invite experienced psychological consultants, psychotherapists, and career instructors on campus and outside the school to conduct career selection psychology for students tutoring, etc. [19]. These distinctive, focused, and colorful career choice special education activities can help students understand social dynamics, employment situation, and career characteristics, so as to clarify learning goals, generate learning motivation, adjust career selection mentality, and establish correct career values. Lay a good foundation for a successful career in the future. Alleviate the employment pressure brought by the pressure on students, and ensure that graduates have a mentality to smoothly adapt to the society and enter the society through the holding of various activities and mental health activities. Social practice activities not only give students the opportunity to directly contact the society and enhance their cognition of social life, but also make them better understand all aspects involved in professional life, realize their own shortcomings in the future professional field, and then can better arrange the study and life in school. At the same time, these social practice activities are of great benefit for students to better master the skills they have learned, apply the theories they have learned to work practice, and improve their sense of efficacy in career selection.

### 4.5. Suggestions for Strengthening Mental Health Education

#### 4.5.1. Distinguish Different Types of Psychological Counseling Projects

Individual consultation mainly includes consultation room consultation, telephone consultation, and letter consultation. Consultation in the consultation room means that students come to the consultation room for consultation once or twice a week to solve the confusion and psychological problems in study and life. The consultation room should have a standardized consultation appointment card and consultation record book when consulting and archive it in time after the consultation. When making a consultation appointment, students should first fill in basic information, such as name, gender, age, class, contact information, emergency contact information, and suitable time for consultation. The consultation record manual generally includes consultation instructions, detailed information of visiting students, consultation process records, and consultation conclusion summary. The consultation instructions mainly include the introduction of the consultation room, the rights and obligations of psychological counselors, the rights and obligations of visiting students, the principle of confidentiality, and the right of the consultant to interrupt the consultation. Counseling students should sign their names to agree to counseling after reading these. The record of the consultation process should include the date, brief introduction to the consultation content, and consultation plan. The summary filled out by the psychological counselor at the end of the consultation should include the reasons for the end of the consultation and the effect of the consultation. Filling out the consultation record booklet will help psychological counselors to accurately grasp the mental health status of students, as well as future reference and case studies. The consultation-visit relationship formed by telephone consultation and letter consultation is relatively special. The psychological counselor can only talk to the consultation students by telephone or letter and cannot directly observe other aspects such as the body language of the consultation students. Therefore, special attention should be paid to the content and time of the conversation for the sake of control and other issues and to try to avoid the problem of telephone or letter harassment. The counseling room should arrange a psychological teacher on duty every day and publish the brief introduction, duty time, and consulting telephone number of the counseling teacher on the campus network and the consulting window [20]. Generally speaking, for developmental counseling and preventive counseling due to career choice, either room counseling, telephone counseling, or letter counseling can be used, but if psychological barriers to career choice have occurred, counseling room counseling should be used.

#### 4.5.2. Seize Different Time Periods for Business Management Consulting Services

Although students study in school for a short period of time, their psychological conditions are different in different periods, and their psychological characteristics have obvious stages. Therefore, grasping the different periods of students' psychological development to provide counseling services can play a multiplier effect with half the effort.

The census of freshmen's mental health status has become a must-have in the education of freshmen in various colleges and universities in recent years. Advantages: discover your potential, and find a career path suitable for your own development. During the census of the mental health of freshmen, you should guide students to take relevant career assessments, such as professional personality assessment and Hollander vocational interest assessment. Conditional schools should purchase relevant software to guide students in online assessment, and psychological counselors will also give scientific and reasonable psychological assessment explanations and guidance. Soon after the freshmen enter the school, the school should carry out career education for the freshmen, introducing the development status of the major they are studying, the occupational fields involved, the employment status of the previous students, the subjects to be studied in this major, and the knowledge and skills to be mastered. Wait. It should be combined with career assessment and career education to guide freshmen to establish career goals and carry out career planning [21].

#### 4.5.3. Carrying Out a Number of Activities of Psychological Education Consulting Services for Career Selection

Psychological counseling service agencies for career selection should take the initiative to interview students who have psychological confusion and psychological barriers in career selection based on the problems reflected in the students' psychological files, and provide psychological counseling through meticulous consulting services. At the same time, for students who take the initiative to come to the door for consultation, they should help them in a scientific and orderly manner according to the consultation procedures and methods. For the relevant activities carried out by the school, actively cooperate with and give professional guidance. For the freshman and sophomore groups of students with different majors and different psychological characteristics, the relevant knowledge of career choice and career development will be popularized in different ways, and the occupational psychological quality will be expanded through group training. Compared with nongraduating students, graduating students are a high-risk group of psychological problems when choosing careers. Psychological education counseling service agencies for career selection should work with relevant departments, such as the Employment Guidance Center, to do a good job in the investigation of graduate students' career selection psychology and career selection psychological education, actively carry out consulting services for the problems found in the investigation, and conduct job interviews for students. Psychological counseling refers to teaching students the methods of psychological adjustment when they are frustrated when choosing a career. For students who have had a psychological crisis, the psychological counseling teacher should cooperate with relevant school personnel to rush to the accident site to start work as soon as possible, understand the situation, use professional knowledge to persuade students in psychological crisis in a timely manner, and do a good job of psychological crisis students and surrounding students. Psychological relief work [22]: when the crisis is initially resolved, the guardian should be assisted in further counseling and comforting work, judge whether to refer to a professional institution for treatment based on the actual situation, and cooperate with monitoring and referral. Conditional colleges and universities can set up a psychiatric outpatient clinic in the school hospital or hire a professional psychiatrist to visit the school hospital on a regular basis, which is more conducive to early detection of psychological crisis problems and timely resolution of problems.

## 5. Conclusion

Students' mental health has always been a hot topic in colleges and universities. How to make students integrate into the collective and society faster and better is also one of the most difficult problems for educators. Students want to improve their competitiveness; not only must they have superb professional skills, but they also must have good social adaptability. Only in this way can you quickly complete your identity change and quickly adapt to workplace life. Students' social adaptability is not innate, but gradually formed through long-term positive mental health education. Under this background, it is necessary to formulate a targeted positive mental health education plan according to the actual situation of the students, so as to comprehensively improve the comprehensive quality of students in this way. According to other researches on college students' mental health and social adaptability, they also start with college students' social adaptability to analyze the current situation of college students' social adaptability and mental health. Correlation analysis was carried out on the mental health of college students in four dimensions, and then the prediction degree of social adaptability to mental health was analyzed.

Students' social adaptability has increased. In addition to improving their national society and workplace work, it also plays a role in the conservation of the natural environment. And explore this one theme; just accord with how this special issue wants to explore creativity in environment management.

## Figures and Tables

**Figure 1:** Students' work stress cognitive score.

**Figure 2:** Students' mental health status.

**Figure 3:** The specific relationship between students' mental health states.

**Figure 4:** The specific state of students' mental health.

**Figure 5:** Sources of students' mental health problems.

**Figure 6:** Comparison of public ecological and environmental behaviors in my country.

**Figure 7:** Students' satisfaction with mental health education.

**Table 1:** Statistical table of depression tendency.

Object of investigation	No tendency to depression (0–9 points)	Have a tendency to be depressed (10–16 points)	High risk of depression (17–27 points)
Undergraduate boys	72.6	20.8	6.6
Undergraduate girls	70.0	22.4	7.6
College boys	90.2	8.2	1.6
College girls	89.3	8.8	1.9
National adults (reference)	78.8	16.7	4.5

**Table 2:** Ideological and political education and mental health education.

Subject different points	Ideological and political education	Mental health education
Theoretical basis	Marxism–leninism, lao ledong thought, leng xiaoping theory, and the important thought of “three represents”	Various theories of mental health and counseling and therapy

Purpose	Solve the problems of students' marxist positions, viewpoints, and other political views and high-level social orientation	Optimize psychological quality, develop psychological potential, improve mental health, prevent and cure psychological diseases, cultivate students' sound personality, good personality, improve social adaptability, promote all-round development

Content	Through the education of world outlook, outlook on life, values and patriotism, collectivism, socialist theme education, moral education, situation policy and basic line education to provide spiritual motivation, intellectual support, talent and political guarantee for the socialist cause	Publicize and popularize the knowledge of mental health, introduce the ways to improve mental health, impart the methods of mental health, and analyze the abnormal psychological phenomena

Working principle	Open principle and value-oriented principle	Confidentiality principle and “value neutrality” position

The subject of teaching: role positioning	Teachers are mainly indoctrinated education, and teachers and students are the relationship between education and the educated	Teachers and students often appear in an equal and cooperative relationship, teachers play a catalytic role in the role of supporters and supporters

Evaluation criteria	Measured by the completion of the task and the cohesion of the class, whether the students can be trained as “four have” newcomers and adhere to the right political direction	Whether the negative emotions of the educated have been alleviated, whether the psychological obstacles have been gradually eliminated, whether the mental diseases have been alleviated and cured, whether the ability to adapt to the environment has been enhanced, and so on

## Data Availability

The labeled data set used to support the findings of this study is available from the corresponding author upon request.

## References

[1] Adlington K., Easter A., Galloway H., Howard L. M. (2022). Mental health is neglected in maternal ear miss research. *BMJ*.

[2] Zhang L., O’Malley I., Cruz-Gonzalez M., Sánchez González M. L., Alegría M. (2022). Factors associated with mental health service use among black, latinx, and asian older adults in community-based organizations. *Journal of Applied Gerontology*.

[3] Brewer M. L., Van Kessel G., Sanderson B. (2019). Resilience in higher education students: a scoping review. *Higher Education Research and Development*.

[4] Elimear S., Gogan E., Doyle L., Grainne D. (2021). Decider life skills training as a method of promoting resilience with mental health student nurses on clinical placement. *Nurse Education in Practice*.

[5] Darius S., Bunzel K., Ehms-Ciechanowicz E., Irina B. (2021). Psychische gesundheit bei referendaren mental health among student teachers. *Pravention und Gesundheitsforderung*.

[6] Payne H. (2022). Teaching staff and student perceptions of staff support for student mental health: a university case study. *Education Sciences*.

[7] Sutton H. (2021). Study reveals increase in mental health crises for student-veterans. *Recruiting & Retaining Adult Learners*.

[8] Baber M., Bate W. (2021). Student mental health—a public health challenge?. *Perspectives in Public Health*.

[9] Homer S. R., Solbrig L., Djama D., Anne B., Sarah K., Jon M. (2021). The researcher toolkit: a preventative, peer-support approach to postgraduate research student mental health. *Studies in Graduate and Postdoctoral Education*.

[10] Smith M. L. (2021). Student mental health: a guide for teachers, school and district leaders, school psychologists and nurses, social workers, counselors, and parents. *Health & Social Work*.

[11] Diaz Y., Fenning P. (2021). Toward understanding mental health concerns for the latinx immigrant student: a review of the literature. *Journal of Urban Economics*.

[12] Chaturvedi K., VishwakarMa D. K., Singh N. (2021). COVID-19 and its impact on education, social life and mental health of students: a survey. *Children and Youth Services Review*.

[13] De Jonge M., Sonia J., Guy E. F., Sabiston C. M. (2021). On campus physical activity programming for post-secondary student mental health: examining effectiveness and acceptability. *Mental Health and Physical Activity*.

[14] Lavergne J. A., Kennedy M. L. (2021). Telepsychiatry and medical students: a promising mental health treatment for medical student use both personally and professionally. *Current Psychiatry Reports*.

[15] Bedrossian L. (2021). Prepare for intensifying COVID‐related student suicide risk and mental health needs. *Disability Compliance for Higher Education*.

[16] Shiratori Y., Ogawa T., Ota M. (2022). A longitudinal comparison of college student mental health under the COVID-19 self-restraint policy in Japan. *Journal of Affective Disorders Reports*.

[17] Pankow K., Mchugh T., Mosewich A. D., Holt N. (2021). Promoting mental health in university student-athletes.png. *Psychology of Sport & Exercise*.

[18] Payne H. (2022). Teaching staff and student perceptions of staff support for student mental health: a university case study. *Education Sciences*.

[19] Hou T., Zhang T., Cai W. (2020). Social support and mental health among health care workers during coronavirus disease 2019 outbreak: a moderated mediation model. *PLoS One*.

[20] D’Eon M. F., Thompson G., Stacey A. (2021). The alarming situation of medical student mental health. *Canadian Medical Education Journal*.

[21] Gallea J. I., Medrano L. A., Morera L. P. (2021). Work-related mental health issues in graduate student population. *Frontiers in Neuroscience*.

[22] Gindidis S., Larsen M. (2021). Apps for secondary school student mental health and wellbeing. *Building Better Schools with Evidence-Based Policy*.

